# Toxicity and Antiulcer Properties of *Ipomoea wightii* (Wall.) Choisy Leaves: An *In Vivo* Approach Using Wistar Albino Rats

**DOI:** 10.1155/2022/4328571

**Published:** 2022-05-18

**Authors:** Saikumar Sathyanarayanan, Puthanpura Sasidharan Sreeja, Karuppusamy Arunachalam, Thangaraj Parimelazhagan

**Affiliations:** ^1^Department of Botany, PSG College of Arts and Science, Coimbatore 641014, Tamil Nadu, India; ^2^Bioprospecting Laboratory, Department of Botany, Bharathiar University, Coimbatore 641046, Tamil Nadu, India; ^3^Department of Botany, NSS College, Nemmara, Palakkad, Kerala, India; ^4^Key Laboratory of Economic Plants and Biotechnology and the Yunnan Key Laboratory for Wild Plant Resources, Kunming Institute of Botany, Chinese Academy of Sciences, Kunming 650201, China; ^5^Southeast Asia Biodiversity Research Institute, Chinese Academy of Sciences, Yezin, Nay Pyi Taw 05282, Myanmar

## Abstract

Humans have been using herbs to prevent and cure various ailments since antiquity, and *Ipomoea wightii* is a significant medicinal plant known for its wide ethnobotanical uses. Although the plant is known to treat ulcers, there is no significant scientific validation. The present study aimed to assess the acute toxicity, subacute toxicity, and antiulcer properties of the leaf methanol extract of *I. wightii* (IWL). In the subacute study, the extracts were given orally at 100, 200, and 400 mg/kg doses for 28 days, and we analyzed the biochemical and histological parameters to evaluate the toxicity of IWL. Two different models were assessed to explore antiulcer properties, such as indomethacin- and ethanol-induced ulcer model. Ulcer areas and ulceration percentage histopathology of the stomach were used to study the efficacy of extracts. The acute toxicity study showed that IWL was safe to the maximum dose of 2000 mg/kg body weight. In a subacute toxicity study, the oral administration of IWL did not produce any mortality in the tested animals. The analysis of haematological, liver biochemical, kidney profile, lipid profile, and *in vivo* antioxidant parameters depicted that all the values were within the control limits after the experimental period and were considered nontoxic to animals. Additionally, the antiulcer study demonstrated a positive response of IWL in a dose-related manner (indomethacin- and ethanol-induced models). Macroscopic analysis showed that pretreatment with *I. wightii* leaf methanol extract significantly reduced the gastric lesion and decreased the ulceration area (14.52 mm^2^), demonstrating superior results to the positive control group (27.71 mm^2^). The histopathological analysis revealed that pretreatment with a high dose of 400 mg/kg of *I. wightii* leaf methanol extract and positive control group (omeprazole) markedly protected pathological effects, and the gastric mucosa appeared normal. In conclusion, *I. wightii* has solid nontoxic potential as a promising native herb for an integral therapy for the treatment of ulcers.

## 1. Introduction

In the modern era, plants are the only assuring source for developing medications to treat many diseases [1–4]. More than a few hundred medicinal plants, for-instance *Aglaonema hookerianum* [5]*, Alstonia scholaris* [6]*, Andrographis paniculata* [7]*, Lepidagathis hyaline* [8]*, Ophiorrhiza rugosa* [9]*, Psychotria calocarpa* [10]*, Spirulina platensis* [11], and *Syzygium fruticosum* [12], are widely used as therapeutic sources because of their active principles. India is an ethnobotanically diverse country since traditional medicine relies on ethnic groups for primary health. India has about 35,000 plants, which have several medicinal values, among which 8000 plant species are used in traditional medicine to improve health conditions. However, scientific validation and the effectiveness of many plants have not been well-documented so far [13]. Phytochemicals could be extracted successfully from medicinal plants for a wide range of use as preventive or therapeutic medicine to treat cancer, liver disease, diabetes, and high blood pressure [14].

Plants synthesize a wide variety of metabolites that form complex compounds, such as polyphenols [15], flavonoids [16, 17], furanocoumarins, [18] and coumarins, [19] that may be beneficial to humankind. Most developed nations exert certain regulations and have developed reliable strategies for monitoring the safety and standardization of these products while providing quality assurance for any of such natural substances [20]. However, many traditional and complementary medicine practitioners often refute the WHO certification scheme to regulate the quality of medicinal products [21]. It explains why divergent opinions exist on the various applications of medicinal herbs [22]. Also, it constitutes a setback against the scientific justification of folklore medicines applications [23]. Three crucial steps must be followed to ensure and maintain the quality, efficacy, and safety profile of herbal drugs. Firstly, there must be a study to show the safety profiles of any compound/product that is claimed to be beneficial to a living organism. The second is to assess the chemical constituents of the traditional medicinal agent. Lastly, it is to set the guidelines to investigate the proposed folklore application, which is a step toward drug development and discovery [24, 25]. Therefore, there has been an increased effort to identify herbal-derived therapeutic agents with reduced side effects to treat the ailment. In many eastern countries, traditional medicines in the mode of herbal extracts have been used to treat diseases. On the other hand, herbal medicine can be further examined before their use regarding the toxicity [26].

Gastric ulcer is a severe disease that affects about 5% to 10% of the world's population. Gastric ulcer is caused by injury to the gastrointestinal mucosa by smoking, stress, alcohol consumption, prolonged ingestion of nonsteroidal anti-inflammatory drugs (NSAIDs), gastric acid hypersecretion, pepsin activity, gastric contractions, gastric mucosa ischemia, and infection by the bacteria *Helicobacter pylori* [27]. It is well-known that orally consumed ethanol is rapidly absorbed into the bloodstream from the stomach and intestine. A high concentration of ethanol directly destroys the gastric mucosa. Currently, gastric ulcers are managed by chemical and cytoprotective drugs. However, most of these drugs have side effects, such as joint pain, altered heartbeat, hemopoietic changes, gynecomastia, cancer, and systemic alkalosis [28, 29]. The number of plant-derived phytocompounds, such as curcumin [3], cannabidiol [30, 31], and palmitoylethanolamide, [32–34] are used to treat gastric ulcers [30–34]. Similarly, there is a need to search for a plant with a strong traditional and scientific background with antiulcer potential and safety herbal.

*Ipomoea wightii* (Wall.) Choisy belonging to the family Convolvulaceae has long been used in traditional herbal medicine in India and Africa. The family comprises nearly 1600 species that are widely distributed worldwide. It is a perennial herb with twining or prostrate stem from tropical Asia. The leaves were used as a leafy vegetable by Paliyar or Paliyan tribes in Southern India [35]. The ashes of the plant are used to treat leprosy by many. In Rwanda, leaf extracts were taken orally to treat liver complaints, whereas the root is taken against a cough in East Africa, and the leaf was used to treat stomachache and ulcer [36]. In this perspective, *Ipomoea wightii* has immense therapeutic potential, which must be investigated scientifically. With this background and existing meager reports on the scientific evidence of this species, the present study was designed for exploring toxicological profile by acute, subacute toxicity, and antiulcer potential of *Ipomoea wightii* using *in vivo* animal models by the evaluation of haematological, biochemical, and histopathological parameters.

## 2. Materials and Methods

### 2.1. Chemicals

All chemicals, solvents, and reagents used were of the analytical grade and purchased from HiMedia Laboratories Pvt. Ltd., Mumbai, India, and Sisco Research Laboratories Pvt. Ltd., Mumbai, India. Millipore water (Direct-Q3, Millipore, Millipore Corporation, Molsheim, France) with a resistivity of 18.2 ΜΩ·cm at 25°C was used in all analyses.

### 2.2. Collection and Identification of Plant Material

*Ipomoea wightii* (Wall.) Choisy was collected during the month of January 2016 from Anaikatti, Coimbatore district of Tamil Nadu, India. Its authenticity was confirmed by comparing the voucher specimen at the Madras Herbarium (MH) of Botanical Survey of India, Southern Circle, Coimbatore, Tamil Nadu (BSI/SRC/5/23/2016/Tech/74). Furthermore, the voucher specimen (Accession No. 006998) was deposited at the Department of Botany, Bharathiar University, Coimbatore.

### 2.3. Preparation of Plant Extracts and Quantification Phytochemical Analysis

#### 2.3.1. Preparation of Plant Extracts

The collected plant leaf materials were cleaned to remove adhering dust and were dried under shade (room temperature). The leaf samples are powdered using a mixer grinder (Dynamix—750 W, Sujata, Mittal Electronics, New Delhi, India). The powdered leaf materials (100 g) were packed in small thimbles using Whatman No. 1 filter paper (Imperial Scientific Works, Coimbatore, India) and extracted with solvents (500 mL), such as petroleum ether, ethyl acetate, methanol, and water, in the increasing order of their polarity using Soxhlet apparatus. Each time before extracting with the next solvent, the thimble was dried in a hot air oven (New Lab, Newlab Equipments, Coimbatore, India) at 35°C. Based on the activity for further studies, the methanol extract was selected and concentrated in a rotary vacuum evaporator and stored in a deep freezer at −20°C (BFS-150, Celfrost Innovations Pvt. Ltd., Haryana, India).

#### 2.3.2. Quantification Phytochemical Analysis

The phenolics, flavonoids, and tannin contents of the plant extracts were determined according to the method described by Thangaraj [37].

### 2.4. Experimental Animals

Five- to six-week-old female (*n* = 96) Wistar rats (150–200 g) were used for the study. The animals were obtained from the animal house, IRT Perundurai Medical College, Erode, Tamil Nadu, India. The animals were maintained in polypropylene cages with paddy husk bedding at a temperature of 24 ± 2°C, and a relative humidity of 30% to 70% in light/dark cycles of 12 h was followed. All animals were allowed free access to water and fed with standard commercial pelleted rat chaw (M/s. Hindustan Lever Ltd., Mumbai). All *in vivo* experiments were performed after approval with the regulations specified by the Institutional Animal Ethical Committee (Approval Reg. No: NCP/IAEC/2017-18/09), Nandha College of Pharmacy, Erode, Tamil Nadu, India.

### 2.5. Acute Toxicity

Five- to six-week-old Wistar rats (*n* = 6/dose) selected by random sampling technique were employed in this study. The animals fasted for 12 h with free access to water only. The leaf methanol extract of *I. wightii* (IWL) (suspended in distilled water with 0.1% of Carboxymethyl Cellulose (CMC)) was administered orally at a dose of 5 mg/kg initially to rats and observed for 24 h for any mortality. If mortality was observed in 4/6–6/6 animals, the dose administered was considered toxic. However, if no mortality was observed, the extract treatment was repeated with higher doses, such as 50, 500, 1000, and 2000 mg/kg, and observed for mortality. The behavior parameters, such as motor activity, tremor, convulsion, straub reaction, aggressiveness, pilo erection, loss of lighting reflex, sedation, muscle relaxation, hypnosis, analgesia, ptosis, lacrimation, diarrhea, and skin colour, were also observed for the first hour and after 24 h of test drug administration [38, 39]. 1/20^th^, 1/10^th^, and 1/5^th^ of the maximum dose administered (i.e., 100, 200, and 400 mg/kg) were selected to carry out the subacute toxicity and antiulcer study of *I. wightii* leaf methanol extract.

### 2.6. Subacute Toxicity

Five- to six-week-old Wistar albino rats (150–200 g) were divided into five groups of 6 animals each. Group I was considered to be the untreated control (UC), group II was treated with 0.6% CMC and was marked as the vehicle control (VC), and groups III, IV, and V were treated with a different concentration based on the acute toxicity results of (100, 200, and 400 mg/kg p.o) *I. wightii* leaf methanol extract. They were considered to be IWL100, IWL200, and IWL 400. They were fasted overnight and treated as mentioned above by an oral gavage daily for 28 days. Drug administration was terminated on the 28^th^ day, after which the rats fasted for 24 h. On the 29^th^ day, the rats in each group were weighed and anesthetized with pentobarbital sodium, and blood samples were collected for biochemical and hematological analyses. Following sacrifice, a thorough necropsy was performed on all animals, and the organs, such as the liver, spleen, brain, and kidney, were dissected for histopathological investigation.

#### 2.6.1. Body Weight, Organ Weight, Organ Index, Feed, and Water Consumption

The rats were observed twice daily for abnormal clinical signs (general clinical observations). Feed and water consumption were measured daily by weighing the feeders. Body weights were recorded on days 0, 14, and 28. All the organs were examined visibly for any abnormalities in the structure. Necropsy was taken, and selected organs, such as the liver, kidney, brain, and spleen, were dissected and washed thoroughly in ice-cold normal saline, and the weights were recorded. Behavioral manifestations and all observations were systematically recorded for each rat. Weight gained (%) and organ indexes were calculated using the following formula [40]:

(1) $$\begin{array}{c} \text{Weight gained}\left(\%\right)=\frac{\left(\text{Final weight}-\text{Initial weight}\right)}{\left(\text{Final weight}\right)}\times 100,\\ \text{Organ index}=\frac{\left(\text{Organ weight}\right)}{\left(\text{Body weight}\right)}\times 100. \end{array}$$

#### 2.6.2. Haematological Profile

Blood was drawn by puncturing the retro-orbital plexus under anesthesia. Whole blood was collected into bottles containing the anticoagulant and ethylene diamine tetra-acetic acid (EDTA) and analyzed for hematological parameters like the hemoglobin count using a hematology analyzer (model ABX-Micro-S-60). Total white blood cells (WBC) were measured after diluting Turk's fluid blood and counting them using a hemocytometer.

#### 2.6.3. Preparation of Serum from Blood

The blood withdrawn was allowed to clot. The serum was separated by centrifugation at 3000 rpm for 15 min. It was analyzed for various biochemical parameters (liver and kidney profile), including total bilirubin, total protein, albumin, globulin, alkaline phosphatase (ALP), aspartate transaminase (AST), alanine transaminase (ALT), creatinine, bilirubin, and lipid profile, such as total cholesterol (TC), triglycerides (TG), HDL, LDL, and VLDL cholesterol, were determined using Span Diagnostics Limited kit, India [41].

#### 2.6.4. Analysis of Liver Homogenate

The excised liver tissues were homogenized in 10% w/v 0.1 M Tris buffer (pH 7.0) and centrifuged at 14,000 rpm for 10 min. The supernatant was used for the measurement of liver enzymatic and nonenzymatic antioxidants, such as superoxide dismutase [42], catalase [43], glutathione reductase [44], glutathione-S-transferase [45], reduced glutathione [46], glutathione peroxidase, and lipid peroxidation [47], using standard protocols.

#### 2.6.5. Histopathology

Freshly excised liver, kidney, spleen, and brain from each group were washed in saline and preserved in 10% formaldehyde solution for histopathological studies. It was fixed for 12 h using isopropyl alcohol and xylene and was embedded in paraffin for light microscopic study. Paraffin-embedded tissue sections cut at 5 *μ*m thickness were prepared and stained after deparaffination using hematoxylin and eosin stain. The stained sections were examined for histological architecture [25].

### 2.7. Antiulcer Activity of *I. wightii* Leaf Methanol Extract

The antiulcer properties of *I. wightii* were carried out by two different models, such as nonsteroidal anti-inflammatory drug (indomethacin)-induced gastric ulcer and ethanol-induced gastric ulcer demonstrated by Sreeja et al. [48] and Wang et al. [29], respectively. The Wistar albino rats were divided into five groups of six (*n* = 6), each for two models randomly. Group I was considered to be the untreated control (UC), group II was treated with 0.6% CMC and marked as vehicle control (VC), and groups III, IV, and V were treated with different concentrations based on thre acute toxicity results of (100, 200, and 400 mg/kg p.o) the *I. wightii* leaf methanol extract and were considered to be IWL100, IWL200, and IWL 400. When the treatment was over, the animals were sacrificed by an overdose of anesthetic ether, and the stomach was removed, washed in cold saline (0.9%), cut open through the greater curvature and spread for better visualization, and photographed to analyze the lesions. The extent of the lesions was measured in mm^2^. It was expressed in percentage (%) of ulceration in relation to the total area of the corpus using ImageJ (Version 1.45) software. Histopathology of the stomach was also analyzed as per the standard protocol [25].

### 2.8. Statistical Analysis

The results were expressed as mean ± standard error means (SEM). The analysis of variance (ANOVA) and significant difference between the means were determined by the Dunnett test. The levels *p* < 0.001 were considered to be indicative of significance compared to the control group. All the calculations were performed using GraphPad PRISM software, version 6.01.

## 3. Results

### 3.1. Extract Recovery Percentage

Sequential Soxhlet extraction of 100 g of dried powder of parts of *I. wightii* leaf was carried out using petroleum ether, ethyl acetate, methanol solvents, and hot water. The extraction yield depends on the nature and polarity of solvents. Contrasting with the solvents, water gave the highest yield, whereas ethyl acetate gave the lowest amount of extractive in leaf part of the plant. The leaf yielded the highest water extract (20.48% w/w), followed by methanol (15.97% w/w).

### 3.2. Quantification of Phenolics, Flavonoids, and Tannin Contents

The total phenolics, flavonoids, and tannin contents in *I. wightii* extracts were statistically analyzed and shown in Table 1. The methanol leaf extract registered the maximum amount (99.56 mg GAE/g extract) of total phenolics compared to other extracts. Flavonoid content ranged from 144.53 to 266.93 mg RE/g in the leaf. The highest level of flavonoid was observed in the leaf methanol extract (266.93 mg RE/g extract). Among the different solvent extracts, methanol and ethyl acetate extracts obtained significant (*p* < 0.05) amounts of flavonoids. The leaf showed the maximum tannin content in methanol (96.47 mg TAE/g extract) and water (90.48 mg TAE/g extract) extracts compared to other extracts. Petroleum ether extracts revealed a minimum amount of tannin content, which may be because of the lower solubility of these compounds in low polar solvents. Therefore, the presence of high phytochemical content in *I. wightii* leaf methanol extract indicates the existence of antioxidant and pharmacological properties.

### 3.3. Acute Oral Toxicity Study

The methanol extract of *I. wightii* was subjected to an acute toxicity test in Wistar albino rats. The animals were monitored for 24 h after the administration of extracts at 50, 500, 1000, and 2000 mg/kg doses. The parameters involving the general behaviors, such as alertness, grooming, touch and pain response, tremors, convulsions, righting reflex, gripping strength, lacrimation, straub reaction, aggressiveness, piloerection, loss of lighting reflex, sedation, muscle relaxation, hypnosis, analgesia, ptosis, diarrhea, and skin color, were observed. The methanol extract did not cause any mortality up to 2000 mg/kg.

### 3.4. Subacute Toxicity Study

#### 3.4.1. Bodyweight and Food Intake of Rats Treated with *I. wightii* Leaf Methanol Extract

The oral administration of *I. wightii* leaf methanol extract at the doses of 100, 200, and 400 mg/kg body weight for 28 days did not produce any mortality in tested animals. No sign of toxicity was detected during the experimental periods. The body weight and food intake of treated rats were tabulated in Table 2. No significant changes occurred in the body weight and the food intake in rats treated with different oral doses of the IWL extract. The control and treated (400 mg/kg p.o) rats appeared healthy at the end and throughout the 28 days of the study. Bodyweight increased up to 14% to 18%. However, there were no significant changes in the body weight of rats treated subacutely with repeated oral doses of the extract compared to the control group.

#### 3.4.2. Organ Weight and Organ Index of Rats Treated with *I. wightii* Leaf Methanol Extract

The subacute effect of the IWL extract at the doses of 100, 200, and 400 mg/kg body weight on the organ weight relative to the body weight (organ index) in normal animals was depicted in Figure 1. The weight of organs, such as the brain (Figure 1(a)), liver (Figure 1(c)), kidney (Figure 1(e)), and spleen (Figure 1(g)), in the treated rats did not show any significant (*p* < 0.001) difference from the untreated control group. All the values were within the control limits after the experimental period of subacute studies.

#### 3.4.3. Hematological Parameters of Rats Treated with *I. wightii* Leaf Methanol Extract

The values of haematogram are statistically analyzed and tabulated in Table 3. Hematological parameters, such as total hemoglobin, total WBC, total RBC, and platelet count, did not show any biological or statistically significant (*p* < 0.001) differences in untreated groups and IWL extract-treated groups. The percentage of the other leukocyte cells (lymphocytes, monocytes, and eosinophils) was not altered. No statistically significant changes were observed in erythrocyte parameters. This result indicates that *I. wightii* extract at higher concentrations is nontoxic to the hematological system.

#### 3.4.4. Liver Biochemical Marker Enzymes of Rats Treated with *I. wightii* Leaf Methanol Extract

As shown in Table 4, the oral doses of *I. wightii* leaf methanol extract had no noticeable effect on blood serum parameters, with no significant changes detected in the levels of proteins, bilirubin, and liver enzyme. Additionally, the administration of *I. wightii* leaf methanol extract 400 mg/kg did not cause any significant changes in alanine transaminase (ALT) and aspartate transaminase (AST) activities. Thus, the result confirmed that hepatic enzymes were unaltered significantly (*p* > 0.001) by *I. wightii* (100, 200, and 400 mg/kg) doses when compared with the untreated control.

#### 3.4.5. Kidney and Lipid Profile of Rats Treated with *I. wightii* Leaf Methanol Extract

The creatinine and urea levels were not changed in rats administered with 100, 200, and 400 mg/kg of *I. wightii* leaf methanol extract (Table 5). Following a subacute treatment in normal rats, the serum HDL cholesterol, total cholesterol, triglyceride, and LDL cholesterol levels were unaltered in the treated rats. The other biochemical parameters analyzed did not significantly differ from the control group and in group-group comparison.

#### 3.4.6. *In Vivo* Antioxidant Activities of Rats Treated with *I. wightii* Leaf Methanol Extract

The results of enzymatic antioxidant activity, such as SOD (superoxide dismutase), CAT (catalase), GPx (glutathione peroxidase), GR (glutathione reductase), and nonenzymatic antioxidant GSH (reduced glutathione), in the liver are shown in Table 6. The oral administration of *I. wightii* leaf methanol extract at doses 100, 200, and 400 mg/kg did not significantly alter GSH and GR levels in liver tissues. The levels of SOD also did not show a significant difference compared to the control group. The LPO levels increased in the liver of animals administered with 100 and 200 mg/kg extract.

#### 3.4.7. Histopathological Examination of Rats Treated with *I. wightii* Leaf Methanol Extract

The results of histopathology are shown in Figure 2. Histopathology studies revealed that *I. wightii* leaf methanol extract did not cause any damage to the brain, spleen, liver, and kidney (Figures 2(c) (100 mg/kg), 2(d) (200 mg/kg), and 2(e) (400 mg/kg)). The untreated and treated animal's spleen section showed the normal structure (Figures 2(a) and 2(b)). There are many lymphoid follicles, and most of them showed prominent germinal centres. Sinusoidal congestion, lymphtasis, histocytic proliferation, and the sheet of siderophages were also seen. The section of the kidney shows a healthy renal structure. The renal tubules and glomerulus show normal cellularity, and the interstitial tissue was observed normally in the 400 mg/kg leaf methanol extract-treated group (Figure 2(e)). The histology of the liver tissue did not show any damage to the hepatocyte morphology portal triads and venous system. The sinusoidal spaces and Kupffer cells appeared normal. The glial cells indicate healthy brain tissues in both treated and untreated groups. The astrocytes also seemed to be normal (Figure 2(e)). A portion of the cerebellum did not show any abnormality. The stroma shows minimal edema in the treated groups of *I. wightii* leaf methanol extract (100, 200, and 400 mg/kg).

### 3.5. Antiulcer Studies

#### 3.5.1. Indomethacin-Induced Gastric Ulcer in Rats

Macroscopic analysis showed that pretreatment with *I. wightii* leaf methanol extracts significantly reduced the total indomethacin-induced gastric lesion area, as observed in figures 3(a)–3(f), 4(a), and 4(b). The treatment with indomethacin induced multiple macroscopic lesions with irregular sizes and shapes in the gastric mucosa of rats (64.40 mm^2^). As expected, no lesions were detected in the control group mucosa (Figure 3(a)). Interestingly, the animals treated with 400 mg/kg of *I. wightii* showed decreased ulceration area (14.52 mm^2^), which was seen as superior to the positive control group (27.71 mm^2^). Histological analysis confirmed that pretreatment with *I. wightii* prevented indomethacin-induced histological damage in the superficial layers of the gastric mucosa with congestion by HE (Haematoxylin and Eosin) staining (Figures 3(g)–3(l)). We observed the gastric epithelium with an organized glandular structure and normal mucosa and submucosa (Figure 3(g)). Indomethacin-induced gastric damage administration is seen as a disruption of the surface epithelium and significantly high necrotic lesions (Figure 3(h)). The histopathological images of the stomach treated with *I. wightii* illustrated the destruction of the glandular architecture beyond the loss or disorganization of the cellular epithelium, and it was decreased in a dose-dependant manner. Rats pretreated with 400 mg/kg of *I. wightii* resulted in maintaining glandular organization and cellular architecture with no pathological changes (Figure 3(l)).

#### 3.5.2. Ethanol-Induced Gastric Ulcer in Rats

The morphology of the ethanol-induced ulcerated stomach of rats is presented in figures 3(m)–3(r). Ulcer area and ulcerated percentage are depicted in figures 4(c) and 4(d), respectively. In the results, ethanol-induced negative control group (5 mL/kg, p.o.) produced severe gastric lesions, with the ulcer areas of different forms and sizes being dispersed overall stomach surfaces with an area of 17.97 mm^2^. The oral administration of *I. wightii* leaf methanol extracts one hour before ethanol administration significantly inhibited ulcer formation in rats linearly with increasing concentration. The result shows that 100, 200, and 400 mg/kg doses of *I. wightii* significantly (*p* < 0.001) reduced the ulcer area (2.70, 1.46, and 0.56 mm^2^, respectively). *I. wightii* leaf methanol extract at the 200 and 400 mg/kg dose reduced the gastric lesions with only 1.98% and 1.00% ulcer percentage, respectively. In contrast, the ulcer percentage of negative control was higher (18.23%) when compared to the positive control and plant extract-treated group.

In the histopathological analysis (Figures 3(s)–3(x)), the sections of the control group revealed the normal structure of the gastric mucosa of rats (Figure 3(s)). In contrast, ethanol administration caused the complete degeneration of the gastric mucosa, and inflammatory cellular infiltration and congested blood capillaries in the lamina propria were observed in the ulcer group (Figure 3(t)). Pretreatment with omeprazol (Figure 3(u)) and *I. wightii* leaf methanol extract (Figures 3(v)–3(x)) markedly protected against these pathological lesions noticed in the ulcer group, and the gastric mucosa appeared normal with preserved gastric gland cells.

## 4. Discussion

The use of herbal medicine to prevent and cure various ailments has been practiced by humans since antiquity. It was the main source of treatment before the evolution of modern allopathic medicine. From traditional knowledge, it was reported that *Ipomoea wightii* was used to treat leprosy, liver diseases, cough, and stomachache [35, 36]. Even with advances in herbal medicine, medicinal plants continue to be used without any scientific basis and have survived for generations only in terms of their widespread use. However, toxicology studies show that many plants are harmful or even lethal because of their toxicity [49, 50]. Even the most effective traditional plants should not be used as a therapeutic unless their toxic parameters are adequately assessed. A complete scientific toxicology assessment is mandatory for using a plant for its medicinal effects [50]. The present study investigated the toxicity of the IWL extract through *in vivo* biochemical and hematological parameters.

Acute toxicity tests are needed to assess the adverse effects of the plant extract. The data obtained from this study indicated that *I. wightii* leaf methanol extract was safe after the oral administration of 2000 mg/kg without any clinical signs of toxicity. LD_50_ for oral administration in rats was estimated to be more than 2000 mg/kg body weight, which was considered low toxicity by OECD guideline 423 and included in category 5 [51]. The same protocol was followed by Harish [52] to evaluate the toxicity of *I. eriocarpa* whole plant and observed with no mortality, thus corroborating our study. Sireeratawong et al. [53] has clearly explained that the general behavior and body weight alone can determine the toxicity of any compound. Therefore, the results obtained in the acute toxicity assay conformed that leaf methanol extract was nontoxic.

In the subacute toxicity study, no significant difference in body weight was observed at 100, 200, and 400 mg/kg in rats during the 28-day oral administration of IWL extract. According to Feres et al., if 10% of the initial body weight is lost, then that the animal should not survive, which is a sign of adverse side effect [54]. However, the present study shows that no animals lost weight. It can be said that growth retardation does not occur during the continuous doses of the IWL extract. Similarly, changes in organ weight are present in the levels of toxicity in animals, which are immediately determined by toxicity tests. When herbal products are ingested, they can be toxic to vital organs, such as the kidneys, liver, spleen, and brain, because of their different roles in the human body. Based on the findings in body weight and the nonsignificant increase in organ weights and index, it can be said that IWL extract is nontoxic to animals.

The hematological analysis is fundamental because the hematopoietic system is one of the most critical targets for toxic compounds. It provides an important indicator of humans and animals' physiological and pathological status [55]. No mortality was reported in subacute toxicity assessments performed with 100, 200, and 400 mg/kg IWL extract doses. In hematological parameters, rats treated with 400 mg/kg of IWL extract showed an increase in the number of red blood cells and a decrease in lymphocytes (80.17%), with respect to the vehicle control (80.83%). These values are within the normal range. Since the administration of IWL extract does not cause a significant change in the measured hematological parameters compared to the controls, it can be suggested that the IWL extract is nontoxic.

The biochemical evaluations are essential to check for any toxic effects on the liver and kidney function. Serum enzymes, AST, and ALT are considered the essential markers of hepatocellular toxicity, and increased activity indicates damage to this organ [56]. The study results demonstrated that the subacute administration of the IWL extract at 400 mg/kg showed no significant changes in ALP and ALT enzymes in treated rats. These results reveal that the IWL extract is nontoxic to treated animals.

The kidney function is assessed by urea and creatinine levels, and an increase in these markers indicates a negative impact on the kidney function [57]. The level of urea in the 400 mg/kg group shows an insignificant difference concerning the control group. It can be confirmed in the histological analysis of the kidneys of rats treated with 400 mg/kg of IWL extract. The long-term administration of IWL extract did not show any significant difference in total cholesterol (400 mg/kg) in rats. The present results agreed with a previous report by Harish [52] that the petroleum ether extract of *I. eriocarpa* showed no difference in the lipid profile compared to the control group rats.

The increase in LPO is considered an important mechanism of cellular damage resulting from the activity of free radicals. Therefore, the nonmodification of LPO level associated with the increase of antioxidant enzymes has been related to the beneficial health effects since the rise of the antioxidant action promoted by the enzymes can control the production of free radicals [58, 59]. This study observed that the IWL extract did not significantly alter any hepatic enzymatic antioxidant levels, such as SOD, GSH, GST, LPO, and CAT compared to the control group of animals. Results also demonstrate that *I. wightii* did not contribute to oxidative stress since the microscopy observations revealed no sign of abnormalities, lesions or necropsy in the group fed with the methanol extract of *I. wightii* leaf compared to the control group. Also, histological observations revealed no anomalies in the liver, kidney, spleen, and brain of groups fed with plant extract compared to the control. They showed no signs of organ toxicity compared to the vehicle group. Thus, the result indicates that *I. wightii* leaf methanol extract did not cause any toxicity.

Gastric hyperacidity and ulcers are very common, causing tremendous human suffering nowadays. Although prolonged anxiety, emotional stress, hemorrhagic surgical shock, burns, and trauma cause severe gastric irritation, the mechanism is still poorly understood [60]. The maintenance of gastric mucosal integrity under an adverse environment of luminal contents depends on a delicate balance of factors regulating cellular proliferation and cell death [61]. The most common proposed mechanism for the ulcerogenic effect of indomethacin is the inhibition of the gastric cytoprotective mediators, prostaglandins, particularly because of the inhibition of the COX pathway of arachidonic acid metabolism in the excessive production of leukotrienes and other products of 5-lipoxygenase pathway. The suppression of prostaglandins synthesis by NSAIDs (Nonsteroidal anti-inflammatory drugs) results in increased susceptibility to mucosal injury, gastroduodenal ulceration, the reduction of mucosal resistance, and the induction of oxidative stress and inflammatory status [62, 63]. Ethanol consumption is known to be one of many factors responsible for gastric ulcer formation because of the production of oxygen-derived free radicals, such as superoxide anions, hydroxyl radicals, and lipid peroxides [64, 65]. Another important common feature of gastric mucosal injury is acute ethanol ingestion observed in alcoholics, and since available antiulcer agents display many side effects [61], there is a need to develop highly effective and safer antiulcer agents. The present study demonstrated that animals pretreated with *I. wightii* leaf possess a dose-dependent protection ability of mucosal layer damage compared to the negative control rats. Also, it was observed that in reducing the epithelial cells damage, *I. wightii* leaf efficacy was slightly higher than the standard drug. The screening of the plant potential against ethanol and indomethacin-induced damage was observed in this study. The animals treated with *I. wightii* leaf extract before administering ethanol and indomethacin significantly reduced the number of ulcer spots and ulcer index. It may be because of the cytoprotective effect of the extract via an antioxidant effect. The considerable raise in the antiulcer activity of *I. wightii* could be attributed to flavonoids and tannins. It is suggested that these active compounds would stimulate mucous bicarbonate and inhibit prostaglandin secretion and counteract the liberating effect of reactive oxygen in the gastrointestinal lumen [66]. These results suggest a strong base for developing a nontoxic therapeutic agent from *I. wightii* leaf for treating gastrointestinal disorders.

## 5. Conclusion

This study is the first report on the toxicological profile and antiulcer effect of *I. wightii*. The oral acute toxicity study showed that the plant was safe to the high dose of 2000 mg/kg of body weight. There is no noticeable toxicity and adverse effect during the subacute toxicity study. Both toxicology experiments suggested that *I. wightii* leaf methanol extract was nontoxic and safe to experimental animals. The antiulcer investigation explored that the leaf could be a potential source for treating gastric ulcers, and this study confirms the traditional claims on the antiulcer property of this plant. Further research is necessary to explore the effective active constituent and its mode of action formulating these pharmacological properties.

## Figures and Tables

**Figure 1:** Effect of subacute doses of *I. wightii* on organ weight and organ index in rats. UC: untreated control, VC: vehicle control (0.6% CMC), and IWL: *I. wightii* leaf methanol extract. The data represent the mean ± standard error (*n* = 6). Not significantly different at ^*∗∗∗*^*p* < 0.001 when compared to untreated control.

**Figure 2:** Effect of subacute oral doses of *I. wightii* on tissue histopathology with samples stained with hematoxylin and eosin. (a) untreated control, (b) vehicle control (0.6% CMC), (c) *I. wightii* leaf methanol extract (100 mg/kg), (d) *I. wightii* leaf methanol extract (200 mg/kg), and (e) *I. wightii* leaf methanol extract (400 mg/kg). Magnification: 40x.

**Figure 3:** Effect of treatment with *Ipomoea wightii* extract (IWL) on the indomethacin- and ethanol-induced gastric ulcer model in rats. i (a–f) Macroscopic observation of indomethacin-induced gastric ulcer model. ii (g–l) Histopathological observation of indomethacin-induced gastric ulcer model. iii (m–r) The macroscopic observation of the ethanol-induced gastric ulcer model. iv (s–x) The histopathological observation of the ethanol-induced gastric ulcer model. Ulcerated areas are marked by circles and arrow marks. Histopathological sections' magnification: 40x. IWL: *I. wightii* leaf methanol extract.

**Figure 4:** Effect of oral administration of the methanol leaf extract of *I wightii* on induced gastric ulcer. (a) ulcer area, (b) ulcer percentage of indomethacin induced rats. NC: negative control (indomethacin, 30 mg/kg), PC: positive control (omeprazole, 25 mg/kg), IWL: *I wightii* leaf methanol extract, (c) ulcer area, and (d) ulcer percentage of ethanol induced rats. NC: negative control (ethanol 5 mL/kg), PC: positive control (omeprazole, 25 mg/kg), IWL: *I. wightii* leaf methanol extract. The data represent the mean ± standard error (*n* = 6). Significantly different at ^*∗∗∗*^*p* < 0.001 when compared to negative control.

**Table 1:** Total phenolic, flavonoid, and tannin contents of *I. wightii* leaf extract.

Plant extract solvent	Total phenolics (mg GAE/g extract)	Flavonoids (mg RE/g extract)	Tannins (mg TAE/g extract)
Petroleum ether	6.18 ± 2.00^g^	144.53 ± 12.76^g^	2.14 ± 0.39^f^
Ethyl acetate	56.73 ± 1.25^d^	220.53 ± 3.03^c^	39.72 ± 2.87^d^
Methanol	99.56 ± 2.15^a^	266.93 ± 7.26^a^	96.47 ± 3.26^a^
Water	95.30 ± 1.44^a^	174.93 ± 2.57^f^	90.48 ± 1.79^a^

Values are the mean of triplicate determination (*n* = 3) ± standard deviation, GAE: gallic acid equivalents, RE: rutin equivalents, and TAE: tannic acid equivalents. Statistically significant at *p* < 0.05, where ^a^ > ^b^ > ^c^ > ^d^ > ^e^ > ^f^ > ^g^ > ^h^ > ^i^ in each column.

**Table 2:** Body weight and feed consumption of rats treated with *I. wightii*.

Groups and doses (mg/kg p.o)	Body weight (g/rat)				Feed consumption (g/rat/day)		
	0^th^ day	14^th^ day	28^th^ day	Weight gained (%)	0^th^ day	14^th^ day	28^th^ day
UC	175.83 ± 28.71	191.67 ± 25.43	204.17 ± 29.40	14.07 ± 0.85	21.50 ± 3.67	24.83 ± 2.40	25.50 ± 2.43
VC	179.17 ± 24.58	204.17 ± 33.08	219.33 ± 30.41	18.29 ± 0.65	21.17 ± 1.72	24.67 ± 1.51	27.17 ± 2.64
IWL 100	185.83 ± 32.31	200.17 ± 32.22	222.17 ± 30.12	16.72 ± 1.40	21.33 ± 1.75	24.17 ± 1.33	25.50 ± 2.17
IWL 200	182.50 ± 20.92	193.83 ± 23.46	209.17 ± 22.99	12.67 ± 2.02	19.67 ± 1.97	23.17 ± 2.64	26.00 ± 2.83
IWL 400	183.33 ± 20.66	199.33 ± 23.70	219.17 ± 21.71	16.36 ± 1.90	21.17 ± 3.19	23.67 ± 1.86	26.17 ± 2.32

UC: untreated control, VC: vehicle control (0.6% CMC), and IWL: *I. wightii* leaf methanol extract. The data represent the mean ± standard error (*n* = 6). Not significantly different at ^*∗∗∗*^*p* < 0.001 when compared to untreated control.

**Table 3:** Hematology profile of rats treated with *I. wightii*.

Groups and doses (mg/kg p.o)	Total haemoglobin Hb (g/dL)	Packed cell volume PVC (%)	Total WBC count 10^3^/*μ*L	Polymorphs(%)	Lymphocytes(%)	Monocytes(%)	Eosinophils(%)	Total RBCcount10^6^/*μ*L	Plateletcount 10^3^/*μ*L
UC	15.17 ± 0.19	44.75 ± 0.24	14.73 ± 0.62	7.00 ± 0.63	75.50 ± 1.41	4.00 ± 0.58	3.83 ± 0.60	5.64 ± 0.17	743.83 ± 47.89
VC	15.38 ± 0.14	45.92 ± 0.31	13.80 ± 0.54	6.00 ± 0.58	80.83 ± 2.41	4.33 ± 0.84	4.17 ± 0.60	5.96 ± 0.14	804.00 ± 23.27
IWL 100	15.40 ± 0.35	48.72 ± 1.55	13.48 ± 1.04	5.83 ± 0.75	81.00 ± 1.59	4.67 ± 0.88	3.17 ± 0.48	6.14 ± 0.25	796.00 ± 23.33
IWL 200	14.37 ± 0.36	40.73 ± 0.45	12.68 ± 1.98	5.50 ± 0.62	80.83 ± 3.22	4.00 ± 1.03	3.67 ± 0.67	5.80 ± 0.20	809.17 ± 23.41
IWL 400	15.15 ± 0.27	45.65 ± 1.11	13.45 ± 0.78	6.83 ± 0.79	80.17 ± 1.89	3.83 ± 0.60	4.17 ± 0.60	6.08 ± 0.16	780.33 ± 22.30

UC: untreated control, VC: vehicle control (0.6% CMC), IWL: *I. wightii* leaf methanol extract, and RBC: red blood cells. WBC: weight blood cells. The data represent the mean ± standard error (*n* = 6). Not significantly different at ^*∗∗∗*^*p* < 0.001 when compared to untreated control.

**Table 4:** Liver profile of rats treated with *I. wightii*.

Groups and doses (mg/kg p.o)	Bilirubin total (mg/dL)	Total protein (g/dL)	Albumin (g/dL)	Globulin (g/dL)	AST (U/L)	ALT (U/L)	ALP (U/L)
UC	0.48 ± 0.01	6.88 ± 0.11	3.53 ± 0.06	3.35 ± 0.06	249.43 ± 17.37	50.08 ± 6.28	157.07 ± 7.95
VC	0.46 ± 0.02	6.78 ± 0.18	3.50 ± 0.10	3.28 ± 0.09	228.31 ± 9.59	51.77 ± 3.58	159.77 ± 15.15
IWL 100	0.58 ± 0.05	7.02 ± 0.29	3.60 ± 0.15	3.42 ± 0.14	247.25 ± 16.71	52.93 ± 4.44	168.00 ± 9.22
IWL 200	0.51 ± 0.03	6.83 ± 0.17	3.57 ± 0.11	3.27 ± 0.07	235.42 ± 7.91	53.73 ± 4.38	164.95 ± 8.72
IWL 400	0.51 ± 0.02	7.10 ± 0.21	3.75 ± 0.18	3.35 ± 0.07	221.68 ± 16.90	49.25 ± 2.74	168.75 ± 17.68

UC: untreated control, VC: vehicle control (0.6% CMC), IWL: *I. wightii* leaf methanol extract, AST: aspartate transaminase, ALT: alanine transaminase, and ALP: alkaline phosphatase. The data represent the mean ± standard error (*n* = 6). Not significantly different at ^*∗∗∗*^*p* < 0.001 when compared to untreated control.

**Table 5:** Kidney and lipid profile of rats treated with *I. wightii*.

Groups and doses (mg/kg p.o)	Urea (mg/dL)	Creatinine (mg/dL)	Total cholesterol (mg/dL)	Triglycerides (mg/dL)	HDL cholesterol (mg/dL)	LDL cholesterol (mg/dL)	VLDL cholesterol (mg/dL)
UC	55.53 ± 2.73	0.38 ± 0.02	152.22 ± 8.78	144.83 ± 7.96	13.97 ± 0.31	116.87 ± 6.89	21.38 ± 1.92
VC	53.65 ± 5.02	0.39 ± 0.02	158.22 ± 11.57	149.35 ± 8.28	13.17 ± 0.64	118.77 ± 10.54	26.28 ± 1.19
IWL 100	58.30 ± 3.37	0.34 ± 0.03	158.38 ± 9.20	152.80 ± 7.46	15.23 ± 0.31	119.17 ± 8.91	23.98 ± 1.23
IWL 200	61.27 ± 2.38	0.38 ± 0.02	173.07 ± 3.29	151.23 ± 8.25	15.65 ± 1.44	130.15 ± 5.15	27.27 ± 1.57
IWL 400	56.23 ± 3.44	0.35 ± 0.03	165.13 ± 6.05	174.28 ± 5.34	14.93 ± 0.27	124.78 ± 5.92	25.42 ± 1.72

UC: untreated control, VC: vehicle control (0.6% CMC), IWL: *I. wightii* leaf methanol extract, HDL: high-density lipoprotein. LDL: low-density lipoprotein, and VLDL: very low-density lipoprotein. The data represent the mean ± standard error (*n* = 6). Not significantly different at ^*∗∗∗*^*p* < 0.001 when compared to untreated control.

**Table 6:** *In vivo* antioxidant levels of rats treated with *I. wightii*.

Groups and doses (mg/kg p.o)	SOD (U/mg protein)	GSH (nM/mg protein)	GR (nM NADPH consumed/min/mg protein)	GST (nM of CDNB-GSH conjugate formed/min/ mg protein)	GP_X_. (*μ*M of GSH oxidized/min/mg protein)	LPO (*μ*M of malondialdehyde released/mg protein)
UC	1.00 ± 0.02	250.68 ± 1.45	16.55 ± 0.46	30.51 ± 0.56	49.33 ± 0.53	9.13 ± 1.09
VC	1.05 ± 0.14	247.97 ± 0.82	16.35 ± 0.58	30.78 ± 1.79	51.10 ± 1.20	12.06 ± 1.62
IWL 100	0.92 ± 0.11	247.59 ± 0.55	16.05 ± 0.60	23.22 ± 0.59	41.45 ± 1.38	31.62 ± 4.69
IWL 200	1.23 ± 0.09	246.43 ± 0.73	16.19 ± 0.53	26.14 ± 0.82	47.08 ± 2.50	22.65 ± 3.48
IWL 400	1.24 ± 0.06	252.22 ± 1.45	17.29 ± 0.43	30.74 ± 4.28	54.30 ± 0.95	8.15 ± 4.14

UC: untreated control, VC: vehicle control, IWL: *I. wightii* leaf methanol extract, SOD: superoxide dismutase, GSH: reduced glutathione, GR: glutathione reductase, GST: glutathione-S-transferase, GP_x_: glutathione peroxidise, and LPO: lipid peroxidation. The data represent the mean ± standard error (*n* = 6). Not significantly different at ^*∗∗∗*^*p* < 0.001 when compared to untreated control.

## Data Availability

The data used to support the findings of this study are available from the corresponding author upon request (Saikumar Sathyanarayanan: drsaikumars@gmail.com).
